This article has been retracted.

# Knowledge and Behavior toward Venous Thromboembolism Event Prophylaxis and Treatment Protocols among Medical Interns in Riyadh

**DOI:** 10.1155/2022/7191178

**Published:** 2022-07-20

**Authors:** Zohair Al Aseri, Jumanah Meshari Muammar, Najd Fahad Aldakkan, Afnan A. Alhazmi, Hadeel Hamad Albraik, Aeshah Abdullah Alasmari, Lyla Mohammed Ashry, Shaik S. Ahmed, Aamer Aleem

**Affiliations:** ^1^Department of Clinical Sciences, College of Medicine, Dar Al Uloom University, Riyadh, Saudi Arabia; ^2^Departments of Emergency Medicine and Critical Care, College of Medicine, King Saud University, Riyadh, Saudi Arabia; ^3^Department of Family and Community Medicine, College of Medicine, King Saud University, Riyadh, Saudi Arabia; ^4^Department of Medicine, Hematology/Oncology Division (Oncology Center), College of Medicine, King Khalid University Hospital, King Saud University, Riyadh, Saudi Arabia

## Abstract

**Objective:**

This study was aimed at evaluating the knowledge and behavior toward venous thromboembolism (VTE) prophylaxis among medical interns.

**Methods:**

This is a questionnaire-based cross-sectional observational cohort study of medical interns that used a validated questionnaire. The questionnaire comprised of items that assessed behavior, knowledge, and self-assessment of VTE risk factors, diagnosis, and prophylaxis. The study was conducted in Riyadh, Saudi Arabia, from October 2020 till September 2021.

**Results:**

The respondents were 246 medical interns. The overall rate of correct responses to behavior items was 41.82%. The overall rate of correct responses to knowledge items was 47.35%. A total of 61.8% responded negatively to the use of VTE risk assessment guidelines (*p* < 0.0001). For the self-assessment of knowledge of VTE, more than 70% believed they did not have appropriate knowledge, were not prepared to establish the risk of VTE, and were not prepared to provide adequate prophylaxis for VTE (*p* < 0.0001). A high proportion of medical interns (83.3%, *p* < 0.0001) believed they needed further training on this topic.

**Conclusion:**

Participants in this study showed poor knowledge and negative behavior regarding the assessment of risk factors, diagnosis, and prophylaxis of VTE. The majority of participants reported they needed training on this topic. These findings underscore the need for educational programs during undergraduate training and orientation of medical interns for VTE risk assessment, diagnosis, and prophylaxis at the beginning of their internship.

## 1. Introduction

Venous thromboembolism (VTE) is a common clinical condition and comprises of deep vein thrombosis (DVT) and pulmonary embolism (PE). The incidence rates of VTE range from 0.06 to 0.87 per 1000 person-years and are substantially higher in high-income countries [1]. VTE is associated with significant morbidity and mortality and is considered the third leading cause of vascular-associated deaths worldwide, with mortality rates between 19.4 per 100 000 and 32.3 per 100 000 of population [2]. In a recent retrospective epidemiological study, the World Health Organization (WHO) mortality database (USA and Canada, 2000–17) was accessed to examine the prevalence of conditions contributing to PE-related mortality reported on death certificates and found an increase in PE-related mortality rates [3]. The US Center for Disease Control and Prevention considers VTE, especially PE, the most common cause of preventable death in hospitalized patients (US Centre for disease control and prevention, 2021) [4]. In an autopsy study, PE was identified as the cause of death in 108 of 982 autopsy cases (11%) in a hospital with an average autopsy rate of 30% ± 0.07% [5].

VTE can be prevented with appropriate thromboprophylaxis, and the need for thromboprophylaxis is determined by VTE risk assessment looking for the presence of risk factors like recent surgery, trauma, immobilization, heart failure, cancer, pregnancy, hormonal therapy, and history of VTE, using various risk assessment tools [6–8]. Evidence from randomized control studies demonstrates significant mortality reduction, safety, and cost-effectiveness of using VTE prophylaxis in appropriate medical and surgical patients [9–12]. Despite wide dissemination of international guidelines on VTE prophylaxis, data show that thromboprophylaxis is under prescribed or misapplied [13–15]. Lack of awareness among physicians is one of the important reasons behind suboptimal thromboprophylaxis utilization [16]. A cross-sectional study performed to assess the awareness of VTE among internal medicine practitioners demonstrated that many practitioners were uncertain of the risk factors for VTE, and the authors concluded that there is a need for ongoing educational program to increase the practitioners' familiarity with the VTE risk factors [16]. Another study showed that internal medicine physicians had different beliefs about VTE prophylaxis than general surgery physicians.

A higher percentage of internal medicine physicians believed that VTE prophylaxis was not required for independent ambulatory patients [17]. Poor knowledge of VTE prophylaxis was also found in a Chinese study which showed clinicians had a low positive response rate regarding their behavior to VTE prophylaxis. The clinicians who responded to the survey suggested the need for more training opportunities on VTE prophylaxis [18].

As poor compliance with VTE prophylaxis is common leading to increased incidence of VTE, the American Heart Association called for action to prevent VTE. Their policy includes VTE knowledge and risk assessment, better implementation of prophylaxis, and reporting, national tracking, and prevention of VTE events [19].

Lack of knowledge of the risk factors for VTE and relevant guidelines can lead to failure among physicians to implement VTE prophylaxis. No study has evaluated the knowledge and behavior of medical interns regarding VTE prophylaxis in Saudi Arabia. This study was aimed at evaluating the knowledge and behavior toward VTE and thromboprophylaxis among medical interns.

## 2. Methods

This was a questionnaire-based cross-sectional observational cohort study of medical interns in Riyadh, Saudi Arabia, using a questionnaire. The study assessed their knowledge and behavior toward VTE risk assessment, diagnosis, and thromboprophylaxis. Ethical approval was obtained from the institutional review boards (IRBs) of the participating institutions. Our target population was medical interns rotating in different specialties at different hospitals in the city of Riyadh who studied at the colleges of medicine in Riyadh. Interns from other colleges of medicine and health care workers other than interns were excluded. The study was conducted from October 2020 till September 2021, in Riyadh, Saudi Arabia.

The data were collected using a data collection form for the demographic characteristics of the medical interns, with a validated questionnaire to assess the awareness of medical interns about VTE risk assessment, diagnosis, and prophylaxis [20]. The questionnaire comprised 8 items that assessed behavior toward VTE prophylaxis and risk factor assessment using multiple-choice questions with the following possible responses: “always, “often,” “not often,” and “never”; 16 items that assessed knowledge of VTE risk factors and prophylaxis; 4 items for self-assessment of VTE risk stratification, diagnosis, and thromboprophylaxis using multiple-choice questions with the following possible responses: “totally agree,” “somewhat agree,” “neither,” “somewhat disagree,” and “totally disagree”; 3 items for the use of guidelines for VTE risk assessment with “yes” and “no” responses; and 4 items for the self-assessment of VTE risk stratification, diagnosis, and thromboprophylaxis.

Other areas of assessment included general information about VTE. Three items were used for the assessment of knowledge of different methods of thromboprophylaxis and 3 items for the assessment of the diagnostic tools of VTE.

The questionnaire was uploaded to an online survey collection tool, and the link was sent to the colleges of medicine and medical interns across the city of Riyadh by email and WhatsApp. Participation in the survey was anonymous and voluntary.

### 2.1. Statistical Analysis

All data collected were coded in an Excel spreadsheet. SPSS package version 26.0 (IBM Inc., Chicago, USA) was used for data analysis. Descriptive statistics, frequencies, and percentages were used to describe the categorical variables. A nonparametric Pearson's chi-square fitness of test was used to observe the statistical significance of observed categorical binary responses of different items related to VTE prophylaxis. A p value of ≤0.05 was used to report the statistical significance of the results.

## 3. Results

Knowledge and behavior toward VTE prophylaxis were assessed among the 246 medical interns. Out of 8 items that assessed behavior, for only 1 item (“How often do you screen for risk factors for venous thromboembolic disease in your hospitalized patients?”), 59.8% of medical intern's responses were positive (always or often) and 40.2% of responses were “never or not always,” which indicated a significant difference (*p* = 0.002). In addition, for 2 items that assessed behavior, the responses were not significantly different (*p* = 0.444 and 0.524), as the responses (“always or often” and “never or not always”) were almost evenly distributed (47.6% and 52.4%; 52% and 48%). For the remaining 5 items that assessed behavior, the binary responses were highly statistically significant (*p* < 0.0001), as a higher proportion (61.8%, 69.5%, 74.8%, 54.1%, and 64.6%) of medical interns responded with “never” or “not always.” The overall rate of correct responses to behavior items was 41.82%, indicating that medical interns' behavior toward VTE prophylaxis was not at the optimum level (Table 1).

For the 16 items that assessed the knowledge of VTE prophylaxis and risk factor assessment, the medical interns' responses for 6 items were positive for items 1 (70.7%), 2 (56.5%), 4 (72%), 6 (68.3%), 9 (74%), and 13 (57.7%), respectively, as they responded with “totally agree,” which was highly statistically significant (*p* < 0.0001, Table 1). For a total of 5 items, the medical interns' distribution of binary responses of “totally agree” and “somewhat agree or did not agree” was not statistically significant, whereas for the remaining 5 items (2, 4, 6, 7, 12, and), a higher proportion of medical interns (85.8%, 88.6%, 68.3%, 58.5%, and 78.5%) responded with “somewhat agree or did not agree” (Table 1), which was highly statistically significant (*p* < 0.0001). The overall rate of correct responses to the items that assessed knowledge was 47.35% (Table 1).

More than 50% of the medical interns (61.8% and 62.6%) responded negatively (with “no”) to the 2 items related to the use of the guidelines for VTE risk assessment, which was highly statistically significant (*p* < 0.0001). In addition, 58.9% of the interns responded positively (with “yes”) for the item “is there a venous thromboembolic disease risk assessment program (model or tool) for the patients in the hospital you work at?”, which was also statistically significant (*p* = 0.005) (Table 2).

Self-assessment of VTE risk stratification, diagnosis, and thromboprophylaxis was carried out using 5 items, where more than 70% of the interns responded with “disagree and totally disagree” (Table 3), which was highly statistically significant (*p* < 0.0001). A significantly higher proportion of interns (83.3%, *p* < 0.0001) responded with “totally agree” regarding the need for training in the management of VTE (Table 3).

For the two items regarding general information about VTE, approximately 82.1% and 63.8% of medical interns, respectively, responded with “agree,” which was statistically significant (*p* < 0.0001) (Table 4).

For the 3 items for assessment of the diagnostic methods of VTE, 43.5% of medical interns agreed for the use of D-dimer, 29.7% of them mentioned the use of a chest computed tomogram, and 47.6% of them agreed for the use of D-dimer plus Doppler ultrasound as reliable methods for the accurate diagnosis of deep vein thrombosis (Table 4).

For the 3 items used for the assessment of the interns' knowledge of different methods of thromboprophylaxis (Table 4), approximately 61.8% and 86.6% of medical interns responded with “agree” and “disagree,” respectively, whereas for the third item, 72.4% of interns responded positively with international normalized ratio (INR) as the correct response, which was statistically significant (*p* < 0.0001).

## 4. Discussion

VTE risk assessment and risk stratification is the initial step to evaluate the need for thromboprophylaxis and should be performed in all hospitalized patients [6–8, 19]. Numerous studies of VTE prophylaxis in hospitalized patients have shown that VTE prophylaxis is under prescribed or not properly applied [13–15]. Although VTE risk assessment is needed in all hospitalized patients [19–21], many physicians believe that VTE prophylaxis is not required for independent ambulatory patients and, therefore, may not assess for VTE risk in these patients. Although this attitude varies among different specialties, it is more common among internal medicine physicians as compared to surgeons [17–18]. Poor knowledge and behavior of VTE prophylaxis was shown in a Chinese study, and participants showed a low positive response rate regarding their behaviors to VTE prophylaxis. The clinicians who responded to the survey suggested the need for more training opportunities on VTE prophylaxis [19–23].

To our knowledge, no recent study has evaluated the knowledge and behavior of medical interns toward VTE prophylaxis. In many institutions, medical interns are usually involved in the initial patient assessment. Their awareness and attitude may play an important part in VTE risk assessment and prophylaxis, and hence, poor knowledge and awareness of VTE prophylaxis may result in failure to provide appropriate risk assessment and thromboprophylaxis. Our study showed that overall knowledge of medical interns regarding VTE prophylaxis and risk factor assessment was poor. Respondents of the current study also showed a negative attitude toward VTE risk stratification and prophylaxis. Moreover, there was poor knowledge and adherence to the guidelines for VTE risk assessment; few participants knew about the published guidelines or had used one of them. More than half of the participants reported that they were involved in the VTE risk assessment of their patients in their respective departments. This raises the concern that poor knowledge and attitude of medical interns towards VTE prophylaxis may lead to under prescription and increased risk of VTE among hospitalized patients.

Our study findings highlight that majority of the medical interns did not have appropriate knowledge about VTE and were not prepared to establish the risk for VTE or provide adequate VTE prophylaxis to the patients. Nevertheless, most of the respondents reported and agreed that they needed further training on this subject. This deficiency underscores the need for more teaching and training regarding VTE prophylaxis prior to starting the internship.

Bearing in mind the widespread poor knowledge and awareness of physicians regarding VTE prophylaxis as shown in other studies [13–18], our study results are not surprising, especially considering the fact that medical interns are at the beginning of their career in clinical practice. This reflects the deficiency of educational programs at the undergraduate level. The importance of educational programs and lectures has been reported in a previous local study that found that education via didactic lectures improved the knowledge of the participants regarding the thromboprophylaxis guidelines [24–27]. The current study showed that there is area for improvement and enhancement of overall knowledge of medical interns toward VTE risk assessment and prophylaxis. Knowledge of medical students needs to be enhanced by incorporating educational courses about VTE risk assessment, diagnosis, and prophylaxis in the undergraduate curricula. Moreover, medical interns should receive orientation on this subject in the beginning of their internships.

Our study has certain limitations. First, all respondents were only from one city, which may not make our findings generalizable to medical interns elsewhere because of the differences in undergraduate curricula and training. Second, the study did not segregate respondents according to their specialty rotations completed before the survey. Third, the timing of the survey was not at a specific period in the internship year, and respondents were in various stages of their internships, which may have influenced the results as interns in the beginning of the internship are expected to have less knowledge of the topic as compared to those at the end.

## 5. Conclusion

Participants in this study showed poor knowledge and negative behaviors regarding the assessment of risk factors, diagnosis, and prophylaxis of VTE. Majority of the participants agreed that they needed training programs for VTE prophylaxis. Apart from additional educational programs during undergraduate training, medical interns should receive orientation for VTE risk assessment, diagnosis, and prophylaxis in the beginning of their internship.

## Figures and Tables

**Table 1:** Distribution of knowledge and behavior responses toward VTE prophylaxis and risk factor assessment (*n* = 246).

Items regarding behaviour toward VTE prophylaxis and risk factor assessment	No. (%)		*p* value
	Always	Often, not always, never	
How often do you screen for risk factors for VTE in your hospitalized patients?	147 (59.8)	99 (40.2)	0.002
When you are in charge of a hospitalized patient, how often do you consider the possibility of them developing VTE?	117 (47.6)	129 (52.4)	0.444
How often do you ask for a history of deep vein thrombosis in your clinical practice?	94 (38.2)	152 (61.8)	<0.0001
How often do you ask for a history of pulmonary embolism in your practice?	75 (30.5)	171 (69.5)	<0.0001
How often do you suspect a diagnosis of VTE in your clinical practice?	62 (25.2)	184 (74.8)	<0.0001
How often do your hospitalized patients with chronic cardiac or respiratory failure receive pharmacological thromboprophylaxis?	128 (52)	118 (48)	0.524
How often do you suggest the use of a thromboprophylactic measure in patients who require a fixed or mobile splint?	113 (45.9)	133 (54.1)	<0.0001
How often is VTE prophylaxis indicated for a cancer patient?	87 (35.4)	159 (64.6)	<0.0001

Items regarding knowledge about VTE prophylaxis and risk factor assessment	Totally agree	Somewhat agree, disagree, neutral, and totally disagree	*p* value
1. In all hospitalized patients, should the risk for VTE be stratified?	174 (70.7)	72 (29.3)	<0.0001
2. The risk for VTE is similar for all types of scheduled surgery.	35 (14.2)	211 (85.8)	<0.0001
3. The risk of VTE is greater in surgical patients than in nonsurgical patients.	109 (44.3)	137 (55.7)	0.074
4. The risk of VTE is similar in both oncological and nononcological surgery.	28 (11.4)	218 (88.6)	<0.0001
5. Thromboprophylaxis measures are more useful if they are initiated before the surgery starts as compared to postoperative initiation.	111 (45.1)	135 (54.9)	0.126
6. The presence of varicose veins is a risk factor for VTE.	78 (31.7)	168 (68.3)	<0.0001
7. Patients on mechanical ventilation have a higher risk of VTE.	102 (41.5)	144 (58.5)	0.007
8. Patients with stroke are at an increased risk of VTE.	139 (56.5)	107 (43.5)	0.041
9. Patients with multiple fractures are at an increased risk of VTE.	177 (72.0)	69 (28.0)	<0.0001
10. There is a risk of VTE in patients who require immobilization with fixed or mobile splints.	168 (68.3)	78 (31.7)	<0.0001
11. The use of hormonal medication raises the risk of VTE in women.	182 (74.0)	64 (26.0)	<0.0001
12. The use of hormonal medications raises the risk of VTE in men.	53 (21.5)	193 (78.5)	<0.0001
13. There is strong evidence demonstrating that flights longer than 4 hours are a risk factor for VTE.	142 (57.7)	104 (42.3)	0.015
14. The risk of VTE is significantly increased in cancer patients.	117 (47.6)	129 (52.4)	0.444
15. Gender is a risk factor for VTE.	114 (46.3)	132 (53.7)	0.251
16. Do you consider obesity as a risk factor for VTE?	135 (54.9)	111 (54.1)	0.126

VTE = venous thromboembolism.

**Table 2:** Distribution of responses toward the use of guidelines for VTE risk assessment.

Items regarding the use of guidelines for VTE risk assessment	No. (%)		*p* value
	Yes	No	
1. Do you know at least one of the published guidelines to assess the risk of VTE?	94 (38.2)	152 (61.8)	<0.0001
2. Do you use any of the published guidelines to stratify the risk of VTE in your patients?	92 (37.4)	154 (62.6)	<0.0001
3. Is there a VTE risk assessment program (model or tool) for the patients in the hospital you work at?	145 (58.9)	101 (41.1)	0.005

VTE = venous thromboembolism.

**Table 3:** Distribution of responses of self-assessment toward VTE risk stratification, diagnosis and thromboprophylaxis.

Items regarding self-assessment toward VTE risk stratification, diagnosis and thromboprophylaxis	No. (%)		*p* value
	Agree	Disagree	
1. Do you have the appropriate knowledge about VTE?	64 (26.0)	182 (74.0)	<0.0001
2. Are you prepared, in theory, to establish (STRATIFY) the risk for VTE in patients?	41 (16.7)	205 (83.3)	<0.0001
3. Are you prepared, in theory, to diagnose VTE?	51 (20.7)	195 (79.3)	<0.0001
4. Are you prepared, in theory, to provide adequate prophylaxis for VTE in patients?	45 (18.3)	201 (81.7)	<0.0001
5. Do you believe that you need training on the prevention and management of VTE?	205 (83.3)	22 (8.9)	<0.0001

VTE = venous thromboembolism.

**Table 4:** Assessment of responses to general information about VTE, knowledge of different methods of thromboprophylaxis, and diagnostic tools of VTE.

	No. (%)		*p* value
	Agree	Disagree	
1. VTE disease is a clinical entity that includes deep vein thrombosis and pulmonary embolism?	82.1%	17.9%	<0.0001
2. Pulmonary embolism is a cause of mortality in your clinical practice?	63.8%	36.2%	<0.0001
1. Intermittent pneumatic compression of the lower limbs is a useful nonpharmacological measure to prevent deep vein thrombosis?	43.5%	56.5%	<0.001
2. All anticoagulants have the same risk of causing bleeding?	29.7%	70.3%	<0.0001
3. What test do you request for the control of anticoagulant therapy with vitamin K antagonists?	47.6%	52.4%	<0.0001
1. What is the most appropriate tool for identifying a low probability of deep vein thrombosis?	61.8%	38.2%	<0.0001
2. What is the most appropriate tool for the diagnosis of pulmonary embolism?	86.6%	17.4%	<0.0001
3. The use of D-dimer plus Doppler ultrasound is reliable for the accurate diagnosis of deep vein thrombosis?	72.4%	27.6%	<0.0001

## Data Availability

The data used to support the results of this study are available on request from the corresponding author.
